The article "Analyzing the Prevalence of Depression and Anxiety Symptoms Among Relatives of Cancer Patients in Kuwait" was published in 2024. Journal: Cureus.

# Analyzing the Prevalence of Depression and Anxiety Symptoms Among Relatives of Cancer Patients in Kuwait

**DOI:** 10.7759/cureus.56989

**Published:** 2024-03-26

**Authors:** Layal Alqaysi, Ahmad F Alenezi, Khaled Malallah, Ebrahim Alsabea, Mona Khalfan, Anwar Alnouri, Haitham Jahrami

**Affiliations:** 1 Department of Internal Medicine, Ministry of Health, Kuwait City, KWT; 2 Department of Medicine, McGill University, Montreal, CAN; 3 Department of Oncology, Ministry of Health, Kuwait City, KWT; 4 Department of Psychiatry, College of Medicine and Medical Sciences, Arabian Gulf University, Manama, BHR

**Keywords:** gad-7, phq-9, relatives, cancer, anxiety, depression

## Abstract

Introduction: The mental health impact on relatives of cancer patients frequently goes unnoticed and is commonly undervalued. This study aimed to explore how personal factors such as the patient's degree of kin, marital status, cancer stage, and number of diagnosed family members are correlated with the severity of depression and anxiety among relatives of cancer patients.

Method: This self-administered cross-sectional survey was conducted in Kuwait, employing a random sampling method to recruit participants. Depression and anxiety symptoms were assessed using the validated Arabic versions of the Patient Health Questionnaire-9 (PHQ-9) and the Generalized Anxiety Disorder-7 (GAD-7) scale.

Results: The mean age of the relatives of the cancer patients was 38.36 years (±13.44), with a female majority (59.72%). The prevalence of depression in the examined population was 60.1%, with the majority having mild depression (39.3%). On the other hand, the prevalence of anxiety in the same group was 51.2%, with the majority having mild disease (27.5%). Being female and having a cancer patient relative in the metastasis stage put patients’ relatives at a greater risk of depression and anxiety.

Conclusion: The diagnosis of cancer necessitates mental health screenings for patients’ relatives, as findings from our study indicate that these individuals are at a high risk of developing depression and anxiety. Targeted support and referrals to specialists are crucial for mitigating the impact on their well-being.

## Introduction

The impact of cancer on patients' mental health is well documented. A diagnosis of major depressive disorder (MDD) is made in 12.5% of cancer patients, whereas its prevalence in the general population is 3.3%, a percentage that indicates a four times greater risk in the former than in the general population [1]. In general, the prevalence of mood disorders is high [1], and around 11%-23% of cancer patients develop mental health disorders [2].

However, the burden placed on cancer patients' families and caregivers is often overlooked, and its effects on their mental health are underestimated [3]. Using the Hospital Anxiety and Depression Scale (HADS), one study showed that 41% of family members responsible for care displayed symptoms of mild to severe depression, and 20% displayed symptoms of mild to severe anxiety [4]. Although the HADS is a screening tool rather than a diagnostic tool, it suggests that caregivers and family members of cancer patients are at a greater risk of developing depression and anxiety than the 12.5% prevalence of MDD in those patients [4]. Another study showed that caregivers scored higher means on the HADS-Anxiety Scale (A) and HADS-Depression Scale (D) than did the patients they cared for [5]. The same study identified a link between the extent of caregiver burden, hours of caregiving, and the presence of depression and anxiety. The Zarit Burden Interview (ZBI) scale was used to quantify caregiver burden, and the study showed that HADS-A/D scores increased with increasing ZBI scores and more caregiving hours [5].

The article "Analyzing the Prevalence of Depression and Anxiety Symptoms Among Relatives of Cancer Patients in Kuwait" was published in 2024. Journal: Cureus.

In addition, the burden of caregiving is more evident when HADS-A/D scores are compared during caregiving and bereavement. A study conducted in Germany [6] showed that family caregivers had higher HADS-A/D scores while caring for a patient than after the patient passed away. In terms of anxiety, the prevalence decreased from 30% with definite cases of anxiety during caregiving to 15% after the patient passed away. The study also established that family caregivers experienced lower scores for emotional quality of life than did the general population. However, the quality of life did not improve even after the patient's death.

The above figures highlight the significance of caregiving in the development of mental health disorders among family members of cancer patients. Nonetheless, the role of other personal factors [7] has yet to be discovered. To bridge this gap, this study aimed to investigate the presence of depression and anxiety among family members of cancer patients, regardless of the extent of caregiving. It also explored the correlation between a) specific personal factors, such as the patient’s relative status, marital status, cancer stage, and the number of relatives diagnosed with cancer, and b) the associated severity of anxiety and depression. The significance of this study arises from the scarcity of literature in this field and the absence of previous local studies on mental health issues among relatives of cancer patients.

## Materials and methods

Study design

This observational descriptive cross-sectional study was conducted at the Kuwait Cancer Control Center (KCCC), the only institution providing cancer treatment within the State of Kuwait. The research aimed to assess the prevalence of anxiety and depression symptoms among relatives of cancer patients. To achieve this, the validated Arabic versions of the Patient Health Questionnaire-9 (PHQ-9) [8,9] and the Generalized Anxiety Disorder-7 (GAD-7) [10] scales were utilized. These standardized scales are widely used for evaluating the severity of depression and anxiety symptoms, thereby providing valuable insights into the emotional well-being of participants. A significant correlation between PHQ-9 and GAD-7 scores (r = 0.8, P < 0.001) was observed.

The article "Analyzing the Prevalence of Depression and Anxiety Symptoms Among Relatives of Cancer Patients in Kuwait" was published in 2024. Journal: Cureus.

Generalized Anxiety Disorder (GAD-7) scale

The Generalized Anxiety Disorder (GAD-7) scale is a self-administered questionnaire used for screening and measuring the severity of generalized anxiety disorder [10]. Consisting of seven items, the GAD-7 assesses the frequency of symptoms associated with anxiety, such as feeling nervous/anxious, not being able to stop worrying, and having trouble relaxing over the last two weeks. Each item is scored from 0 (not at all) to 3 (nearly every day), with the total score ranging from 0 to 21. Scores of 5, 10, and 15 represented the cutoff points for mild, moderate, and severe anxiety, respectively. The GAD-7 has been validated in various populations and is a reliable tool for detecting the presence and severity of generalized anxiety disorder. The GAD-7 scale demonstrated high internal consistency, as indicated by a Cronbach's alpha value of 0.91.

Patient Health Questionnaire (PHQ-9) scale

The Patient Health Questionnaire (PHQ-9) is a multipurpose instrument for screening, diagnosing, monitoring, and measuring the severity of depression [8]. It incorporates the Diagnostic and Statistical Manual of Mental Disorders IV (DSM-IV) depression diagnostics into a brief self-report tool. The PHQ-9 consists of nine items that correspond to the criteria used for diagnosing depressive disorders. Each item is scored on a scale from 0 (not at all) to 3 (nearly every day) to reflect the frequency of symptoms experienced over the past two weeks. The total score ranges from 0 to 27, and depression severity is categorized as none (0-4), mild (5-9), moderate (10-14), moderately severe (15-19), or severe (20-27). This scale has been extensively used in different settings and populations due to its efficacy and reliability in identifying and quantifying the severity of depression. Cronbach‘s alpha of the PHQ-9 scale in the present study was 0.88, suggesting high internal consistency.

Setting, participants, and data collection

The study was conducted between November 21, 2023, and December 21, 2023. Data collection involved the in-person distribution of a survey to eligible participants. Prior to commencing the survey questionnaire, electronic consent was obtained from participants after they reviewed the introductory explanation and agreed to the outlined terms. No personal information was required from participation to ensure anonymity and confidentiality.

The article "Analyzing the Prevalence of Depression and Anxiety Symptoms Among Relatives of Cancer Patients in Kuwait" was published in 2024. Journal: Cureus.

The study included relatives of cancer patients who were 18 years of age or older, with the questionnaire distribution occurring in person. The term "relatives" encompassed individuals such as mothers, fathers, siblings, spouses, sons, and daughters. Exclusion criteria were set to omit individuals under the age of 18 and those who were not relatives of a cancer patient.

Ethical consideration

The research adhered to the ethical principles established by the 1964 Helsinki Declaration and its subsequent revisions. Ethical approval was obtained from the Medical and Health Research Committee of the Kuwaiti Ministry of Health (Approval No: 2240/2023) to execute the present cross-sectional study. Participation in the study was entirely voluntary, and the participants retained the right to withdraw from the study at any stage. To obtain informed consent, a concise and straightforward description of the study objectives was provided in simple nonmedical language within the introduction.

Statistical analysis

The statistical analyses were conducted using R software for statistical computing, version 4.0.3. [11] The chosen significance level was established at 5%, as it denoted the threshold for determining statistical significance. A summary of the statistics was provided for continuous variables, including the mean and standard deviation. For categorical variables, the statistics included the frequency and percentage. An analysis was performed to compare categorical variables, as well as PHQ-9 and GAD-7 scores, across two groups. This analysis used independent sample t-tests or one-way analysis of variance (ANOVA).

## Results

Characteristics of cancer patients’ relatives

The mean age of the cancer patients’ relatives was 38.36 years (±13.44). The majority were female (59.7%) and married (63%). The Kuwaiti population represents 75% of the studied population. As Table 1 illustrates, almost half of the cancer patients had more than one relative diagnosed with cancer (52.1%).

**Table 1:** Characteristics of cancer patient relatives

Characteristics	N (%) or mean ± SD
Age, years	38.36 (±13.44)
Gender	
Female	126 (59.72%)
Male	85 (40.285%)
Nationality	
Kuwaiti	159 (75.36%)
Non-Kuwaiti	52 (24.64%)
Marital status	
Married	133 (63.03%)
Single	66 (31.28%)
Divorce	9 (4.27%)
Widowed	3 (1.42%)
Do you have more than one relative with cancer	
Yes	110 (52.13%)
No	101 (47.87%)
Relationship with the person who has cancer	
Parent (father/mother)	69 (32.70%)
Sibling (brother/sister)	31 (14.69%)
Spouse (husband/wife)	23 (10.90%)
Son/Daughter	6 (2.84%)
Other	82 (38.86%)

Characteristics of patients with cancer

The three most frequent types of cancer among the patients were breast cancer (39.34%), colorectal cancer (16.11%), and hematological cancer (6.64%). Most of the patients had stage IV cancer (metastasis), with 28.44%, while the remaining patients (49.29%) were receiving combined medical treatment (Table 2).

The article "Analyzing the Prevalence of Depression and Anxiety Symptoms Among Relatives of Cancer Patients in Kuwait" was published in 2024. Journal: Cureus.

**Table 2:** Characteristics of the cancer patients

Type of cancer	
Breast cancer	83 (39.34%)
Colorectal cancer	34 (16.11%)
Hematological cancer	14 (6.64%)
Brain cancer	11 (5.21%)
Lung cancer	10 (4.74%)
Lymphoma	10 (4.74%)
Other	49 (23.22%)
Stage of cancer	
Stage I	43 (20.38%)
Stage II	51 (24.17%)
Stage III	57 (27.01%)
Stage IV	60 (28.44%)
Type of treatment	
Radiation therapy	15 (7.11%)
Chemotherapy/Immunotherapy	63 (29.86%)
Oral treatment	29 (13.74%)
Multiple modalities	104 (49.29%)

Frequency of depression and anxiety

A total of 60.1% of the participants in the study group experienced depression. The majority (31.8%) had mild depression, while only 3.8% had severe depression. In comparison, the prevalence of anxiety within the same cohort was 51.2%, with a significant portion (27.5%) having mild anxiety and a notable 10% experiencing a severe form of the condition (Table 3).

**Table 3:** Depression and anxiety severity PHQ-9: Patient Health Questionnaire-9, GAD-7: Generalized Anxiety Disorder-7.

PHQ-9	N (%)
Mild depression	67 (31.8%)
Moderate depression	35 (16.6%)
Moderately severe depression	18 (8.5%)
Severe depression	8 (3.8%)
GAD-7	N (%)
Mild anxiety	58 (27.5%)
Moderate anxiety	29 (13.7%)
Severe anxiety	21 (10%)

PHQ-9 and GAD-7 scores

The mean PHQ-9 score of the cancer patients’ relatives was 7.40 ± 6.28 for females and 6.46 ± 5.58 for males, and this score indicated a mild burden of depression (PHQ-9 5-9), with no significant difference in depression severity by sex, with a P value of 0.267 (Table 4). On the other hand, the mean GAD-7 score was 6.52 ± 5.87 for females and 4.88 ± 4.14 for males, indicating that they experienced mild anxiety as well. However, the association between being female and the severity of anxiety, with a notable P value of 0.027, was a statistically significant indicator (Table 5). In addition, there was a significant difference between cancer stage and depression severity, with a P value <0.05. The mean PHQ-9 score of cancer patients who were relatives who had metastatic cancer was 8.60 ± 5.98, which was greater than that of nonmetastatic cancer patients (Table 4). However, no significant difference was found between cancer stage and anxiety severity, with a P value >0.05 (Table 5).

The article "Analyzing the Prevalence of Depression and Anxiety Symptoms Among Relatives of Cancer Patients in Kuwait" was published in 2024. Journal: Cureus.

**Table 4:** PHQ-9 mean scores for the different domains related to the properties of cancer patients’ relatives PHQ-9: Patient Health Questionnaire-9.

PHQ-9	P value	Mean ± SD
Gender	0.267	
Male		6.46 (±5.58)
Female		7.40 (±6.28)
Nationality	0.411	
Kuwaiti		6.82 (±5.86)
Non-Kuwaiti		7.62 (±6.47)
Marital status	0.492	
Married		6.48 (±5.68)
Unmarried		8.02 (±5.54)
Cancer stage	0.018	
First		5.84 (±5.27)
Second		7.78 (±6.44)
Third		5.56 (±5.79)
Fourth		8.60 (±5.98)
Treatment type	0.441	
Multiple modalities		6.98 (±6.15)
Radiotherapy		9.73 (±8.29)
Oral treatment		5.97 (±4.90)
Chemotherapy/Immunotherapy		6.92 (±5.55)

**Table 5:** GAD-7 mean scores for the different domains related to the properties of cancer patients’ relatives GAD-7: Generalized Anxiety Disorder-7.

GAD-7	P value	Mean ± SD
Gender	0.027	
Male		4.88 (±4.14)
Female		6.52 (±5.87)
Nationality	0.116	
Kuwaiti		5.53 (±5.86)
Non-Kuwaiti		6.87 (±5.88)
Marital status	0.210	
Married		5.46 (±4.97)
Unmarried		6.73 (±4.77)
Cancer stage	0.059	
First		5.51 (±4.46)
Second		6.20 (±5.29)
Third		4.46 (±5.16)
Fourth		7.17 (±5.72)
Treatment type	0.734	
Multiple modalities		5.70 (±5.21)
Radiotherapy		7.40 (±5.77)
Oral treatment		5.48 (±5.38)
Chemotherapy		5.94 (±5.33)

## Discussion

Cancer is a leading cause of death worldwide. It is responsible for one in every six deaths in 2022 [12]. Multiple studies [13-15] have been conducted to highlight the burden of cancer diagnosis, treatment, and progression on caregivers’ mental well-being. The current study investigated anxiety and depression in cancer patients' relatives to determine their prevalence and establish a causal relationship with several factors.

A previous study conducted in Kuwait [16] analyzed the prevalence of psychiatric illnesses among 1,046 primary clinic attendees. The depression and anxiety rates were 22.9% and 17.7%, respectively. In this study, our findings indicate that the prevalence of depression and anxiety among 211 family members of cancer patients is 60.1% and 52.2%, respectively. This significant disparity underscores that being a family member of a cancer patient increases the risk of developing depression and anxiety nearly threefold compared to the general population. This finding is consistent with the findings of other international studies on relatives of cancer patients. For example, studies conducted in Turkey [17], Korea [18], and Taiwan [19] revealed that the prevalence of depression was greater in cancer patients’ relatives than in the general population. On the other hand, studies in Iceland [4] and Norway [20] showed that the prevalence of both anxiety and depression was greater. A meta-analysis study included 30 cross-sectional studies [21] also found a higher prevalence of depression and anxiety among cancer patient's relatives.

The article "Analyzing the Prevalence of Depression and Anxiety Symptoms Among Relatives of Cancer Patients in Kuwait" was published in 2024. Journal: Cureus.

Given that women are approximately twice as likely as men to experience depression and anxiety disorders [22], we considered gender a potential risk factor. In this study, significant gender differences were detected in the prevalence of depression only, with females at a greater risk of depression than of anxiety. However, many studies worldwide have reported different conclusions regarding sex as a risk factor. For example, in Norway [20], a study showed that being a female caregiver for a cancer patient placed you at a higher risk of anxiety, while both genders had almost the same risk for depression. Similar results were reported in studies conducted in Iceland [4] and Iran [23]. On the other hand, a Jordanian study [24] suggested that there was no relationship between gender and examined psychiatric illness. A German study performed on palliative patients and their caregivers suggested that gender had no impact on the psychological well-being of cancer patients’ relatives [6].

The majority of studies show that having a relative diagnosed with cancer is a strong risk factor for depression and/or anxiety. Some of these studies argue that being married to a cancer patient is associated with a greater risk of anxiety [18,25]. Others have identified a positive correlation between anxiety and depression along with a low level of education, low income, and advanced stages of the disease [26]. In contrast, a Turkish study [17] revealed no effect of education level, income, or marital status on depression. In a Ugandan study [27], a strong association was established between anxiety and depression and the relationship with the patient, while no associations with age, education level, employment, marital status, or period of care were detected. This finding highlights the importance of individualizing the chosen risk factors according to the examined population due to differences in culture, level of care, financial status, and average age of the population.

We can observe the variation of findings in different studies and countries. Even within different regions of the same country, certain criteria can be considered risk factors in one area but not in another. This variation needs further explanation in a study that addresses the contributing factors and the nature of each population with respect to their culture and bonds. For this purpose, we recommend further studies that are individualized and/or designed for each country or region in relation to cultural, educational, and income differences. This could help in identifying the risk factors that could be more strongly associated with relatives of cancer patients and the prevalence of mental health disorders.

The article "Analyzing the Prevalence of Depression and Anxiety Symptoms Among Relatives of Cancer Patients in Kuwait" was published in 2024. Journal: Cureus.

Although the current study employed a rigorous methodology, it encountered several limitations. One of the main constraints was the small sample size, resulting from the limited availability of cancer centers in Kuwait. The issue was further compounded by a considerable number of cancer patients receiving treatment abroad, highlighting the necessity for more extensive data collection. These factors collectively could limit the generalizability of our findings.

## Conclusions

The diagnosis of cancer impacts not only patients but also their relatives. Our study shows that the prevalence of anxiety and depression among relatives of cancer patients is almost three times higher than in the general population. This makes mental health screenings critical for physicians to consider for depression and anxiety among family members. By providing counseling, offering diverse treatment options, and facilitating referrals to psychiatric specialists, healthcare providers can substantially mitigate the effects on the mental well-being of patients’ relatives. Further research is recommended with larger sample sizes to enhance the robustness of the findings. Additionally, exploring other risk factors that could contribute to the increased prevalence of depression and anxiety among relatives of cancer patients is advised to provide a more comprehensive understanding of the issue.
